The article "A Deep Learning Approach for Recognizing the Cursive Tamil Characters in Palm Leaf Manuscripts" was retracted in 2023. Reasons: unreliable results or conclusions; concerns about the data; concerns about the results or conclusions; concerns about the peer review.

# A Deep Learning Approach for Recognizing the Cursive Tamil Characters in Palm Leaf Manuscripts

**DOI:** 10.1155/2022/3432330

**Published:** 2022-03-11

**Authors:** Gayathri Devi S, Subramaniyaswamy Vairavasundaram, Yuvaraja Teekaraman, Ramya Kuppusamy, Arun Radhakrishnan

**Affiliations:** ^1^School of Computing, SASTRA Deemed University, Thanjavur 613401, India; ^2^Department of Electronic and Electrical Engineering, The University of Sheffield, Sheffield S1 3JD, UK; ^3^Department of Electrical and Electronics Engineering, Sri Sairam College of Engineering, Bangalore City 562 106, India; ^4^Faculty of Electrical & Computer Engineering, Jimma Institute of Technology, Jimma University, Jimma, Ethiopia

## Abstract

Tamil is an old Indian language with a large corpus of literature on palm leaves, and other constituents. Palm leaf manuscripts were a versatile medium for narrating medicines, literature, theatre, and other subjects. Because of the necessity for digitalization and transcription, recognizing the cursive characters found in palm leaf manuscripts remains an open problem. In this research, a unique Convolutional Neural Network (CNN) technique is utilized to train the characteristics of the palm leaf characters. By this training, CNN can classify the palm leaf characters significantly on training phase. Initially, a preprocessing technique to remove noise in the input image is done through morphological operations. Text Line Slicing segmentation scheme is used to segment the palm leaf characters. In feature processing, there are some major steps used in this study, which include text line spacing, spacing without obstacle, and spacing with an obstacle. Finally, the extracted cursive characters are given as input to the CNN technique for final classification. The experiments are carried out with collected cursive Tamil palm leaf manuscripts to validate the performance of the proposed CNN with existing deep learning techniques in terms of accuracy, precision, recall, etc. The results proved that the proposed network achieved 94% of accuracy, where existing ResNet achieved 88% of accuracy.

## 1. Introduction

For future generations, knowledge from many academics was conserved in both written and oral forms. India went through several ages of speech, drawing, and painting. Writing evolved from drawing through a sequence of natural steps [1]. Different sorts of writing resources, such as leaves, wood, stones, barks, metals, and so on, were found as writing increased. Palm leaves were frequently employed among all accessible materials due to their abundant availability and ability to endure harsh preparing. Palm leaf scripts are an important component of India's written history [2–4]. Palm leaf manuscripts in various Indian languages and written scripts may be found all across the nation in temples, libraries, and museums. An average life of Palm leaves has 300–400 years, despite their conditioning capabilities and many processing, preservation, and conservation procedures. Numerous palm leaf manuscripts written three centuries ago are now in a state of deterioration, and we risk losing the rich material contained on them [5]. These valuable manuscripts provide in-depth knowledge of Astronomy, Literature, Ayurveda, Construction, and Fine Arts written in many vernaculars and scripts from diverse times. In ancient times, the only method to repair and convey this precious material to future age group was to rewrite it. Digitization is being utilized to generate digital pictures of texts to preserve their information as technology advances.

Tamil is among the world's oldest and most recognized languages, having a rich literary heritage. In the ancient period, poets employed Palm leaves, notably in Tamil Nadu, to conceal information [6]. Sangam literature, masterpieces, Vaishnava, Saiva, medicinal works, gastronomy, astrology, Vaastu, gems, music, dance and theatre, and Siddha are all included in the ancient literature. The value of ancient medical texts in Tamil, as well as the necessity to preserve them, has piqued the interest of numerous academics in the recent decade [7]. The conserved old medical writings in Tamil by saints such as Agathiyar were generated for the first phase of a digitalization process to preserve medical materials, and around 10,000 manuscripts were successfully scanned [8]. For digitizing historical documents, handwritten character identification apps used three key methods: statistical, structural or syntactic, and neural network-based techniques.

Optical Character Recognition (OCR) is a method for converting various sorts of documents, such as scanned papers. This method can be classified as either offline or online. Offline handwriting recognition often uses a scanner to acquire the writing optically, and the entire writing is provided as an image [9–11]. Because the characters are identified as they are written, online handwriting recognition is also known as real-time recognition. Online OCR employs pen-based input devices to record the sequence of coordinate points as the character is typed [12]. Handwritten character recognition becomes complex due to various variations in the shape of characters, different writing styles, and overlapping and interconnection of neighboring letters. It also depends on the individual because we do not write the same character in the same manner. It is challenging to create an OCR system with good recognition accuracy for Tamil script [13]. The primary goal of this method is to detect Tamil cursive letters in palm leaf manuscripts. This is accomplished by categorizing the characters into relevant categories based on characteristics collected from each one. The steps below will assist in achieving greater accuracy.

- Image Preprocessing
- Feature Extraction
- Segmentation
- Classification using CNN.

The leaf characters are segmented by using text line slicing, where noises are removed, and morphological operations are carried out in the work. Finally, the palm leaf characters are classified by using CNN model. The experiments are conducted on the collected dataset by using various parameter metrics. The remaining paper is organized as follows: Section 2 consists of Literature Review. The proposed methodology is presented in Section 3. The validation of projected methodology along with existing techniques on the collected cursive Tamil palm leaves manuscripts is presented in Section 4. Lastly, the research work conclusion with its future work is given in Section 5.

## 2. Literature Review

Tamil, one of the world's oldest languages, is gaining popularity among scholars throughout the world due to its historical relevance and capacity to persist for centuries. Individual interests and ideologies of academics have shaped study on palm leaves manuscripts in Tamil poetry over the periods and in a variety of ways. The most prevalent topic of research in the actual world is cursive character recognition of ancient Tamil characteristics, and it focuses on the documentation of Tamil characters to guarantee that a large amount of data is gathered. However, due to improper care, palm leaf manuscripts have been destroyed, as numerous people held them by default. As a result, a rigorous examination of Tamil palm leaf texts, translation, and cataloguing of their publishing were necessary. Thousands of palm leaf texts exist in the hands of institutes and specific healers, but they must be digitized, and proper catalogues were developed for the future. Similarly, numerous researches on the cursive handwriting recognition of the Tamil language are included in the survey. There is, however, no universal technique for identifying cursive Tamil letters (with sufficient accuracy) in their whole. As a result, various approaches have been used in each stage of the recognition process.

As such, this work is one of the first attempts to build cursive training datasets by manual and automated segregation of Tamil palm leaf scripts. Future researchers could make use of the data set to develop expert systems that could then be used for a range of purposes, such as a character classification founded on the period they have changed and the documentation of extinguished characters, and the documentation of characters whose shape could have altered. The study aimed to separate old Tamil palm leaf writings to provide a huge quantity of information about the cursive Tamil character. There have been no previous investigations on the identification of cursive characters in Tamil palm leaf texts. The ThimuNet of CNN is used in this research project to classify cursive Tamil characters, and its performance is confirmed. In the future, the produced training data might be utilized as input and fed into other deep learning systems for further categorization and finding of the cursive letters contained in manuscripts written in Tamil.

Ali and Joseph [8] developed a CNN perfect for dispensation real-time input pictures including Malayalam characters and the job of segmenting words and typescripts from an image and attractiveness prediction using the CNN model. The feature extraction job in this model is done implicitly in CNN by the gradient descent technique. This technique is efficiently utilized for digitizing Malayalam script, which comprises 36 consonants and 13 vowels, is approved out in stages, and has obtained an accuracy of 97.26 percent for the training dataset.

Balakrishnan and Pavithira [9] suggested a method for optimizing CNN using Simulated Annealing, demonstrating the efficiency of character appreciation. They discussed several deep learning approaches, the capabilities of CNN, and ways for training CNNs. According to the definition, “character recognition is the process of classifying and distinguishing characters in an input picture and converting them to ASCII or any similar machine-accessible form.” The suggested approach assessed the OCR accuracy of multiple language texts from numerous books, revealing that the accuracy of CNN by SA is higher than the unique CNN.

Hossian and Afrin [10] provided TEMPLATE MATCHING, a method for extracting characteristics from pictures and identifying precise characters to generate written documents. They claimed, “OCR operates similarly to the human capacity to read.” The picture glance at by the scanner will be the source for the OCR scheme in the same manner as an image viewed by human eyes is the source for the brain in the natural process.” They said that this methodology works by comparing the picture's derived image characteristics and the template for each conceivable displacement. Techniques for word identification and finding in images and videos may be classified as connected component-based methods and texture-based methods. We informed numerous ideas regarding Template Matching, OCR, and the many stages required in Template Matching implementation. They tested the scheme by associating the outcomes of taught datasets to those of unprepared datasets, with accomplished datasets providing 100% accuracy.

According to Baskar [11], the palm leaf was a frequent writing material in primeval India, with the most basic surviving specimens. Furthermore, beginning in the sixth century, the Palmyra palm was employed for document production. Analysts and preservationists have recently been interested in the preservation of records and texts. There has been some awareness in this respect, and their preservation is important. There was a separate custom for palm leaf manuscripts, in which old texts that had become irreversible had to be encrypted on fresh leaves, and the old ones were disposed of in a river. Furthermore, religious laws prohibited pundits from deporting the manuscripts to secure detention facilities. Lack of finances, insufficient apparatus, resources, and qualified staff in document sources are the mechanisms that impede effective care of palm leaf works.

Sageer and Francis [14] suggested a digital library for rare texts as a method for preserving palm leaves. The rate of deterioration to endangered records is higher in a variety of ways, and such leaflets are typically not constrained to the limited bounds of traditional library schemes. They are more commonly found in private groups, official records, and institutional collections. The risk of harm is greater with private groups. Making a digital assortment for endangered materials significantly alleviates this situation. This research examines the different procedures of creating a digital archive for endangered materials and user attitudes toward usability; it focuses especially on user attitudes toward the digitization of palm leaf manuscripts.

According to Devika and Vijayakumar [12], traditional wisdom helps establish long-term interactions between humans and nature. The purpose of this study was to differentiate the contents of palm leaves that can be digitized, the details for digitization, and the various techniques of scanning a palm leaf document. Statistical techniques were used to analyze the collected data. The study provides useful information on the current collection of palm leaf organizations in Tamil Nadu, such as public libraries and private organizations, and nongovernmental administrations. It is critical to have a sufficient quantity of knowledge on the various approaches offered in Tamil Nadu's palm leaf library. This study indicated that manuscript conservation by digitalization is one of the most successful and helpful approaches; however, it is time-consuming and expensive.

Various knowledge schemes were documented in ancient India using palm leaf scrolls, according to Narenthiran and Ravichandran [13]. The wisdom was primarily conveyed through the traditional Sanskrit language in various scripts. This study is based on five document libraries in Tamil Nadu, which are a mix of libraries of varying statuses with superior manuscripts. This research concentrated mostly on the cataloguing of manuscripts and the operations associated with digitalized these archives. The study was based on a national goal, and the papers were recognized.

Sabeenian et al. [15] evaluated localized binarization techniques on Tamil palm leaf scripts, which were recorded to hold a huge quantity of info that is highly useful in everyday life. To protect the data on the palm, digital pictures of each leaf were evaluated and preserved. When necessary, these pictures can be accessed. However, the storage volume required for each leaf is considerable, which raises the cost. These pictures must be binarized in order to acquire only the segmentation and storage. Several computer scientists have been stymied by poor reported picture binarization. This research focuses on palm leaf manuscript pictures that have been binarized using the Sauvola, Niblack, Bradley, and Nick binarization methods.

According to Kiruba et al. [16], one of the most essential phases in manuscript recognition is character segmentation in Tamil palm script. Tamil is India's most frequently used script, and palm scripts contain consonants, modifiers, and vowels. In addition, the accuracy of the recognition approach is influenced by separate letters; therefore, suitable segments are necessary. This paper shows the image segmentation from palm leaf manuscripts of Tamil handwritten letters. The technique consists of three steps: background removal using the Otsu algorithm to separate texts, character segmentation, and line segmentation. This paper proposes a simple histogram-based method for segmenting Tamil palm script characters and discusses many obstacles to Tamil script segmentation.

As Ghosh et al. [17] note out that palm leaf works show a significant role in India's prized national legacy, particularly in relations of their extraordinary accumulation of famous knowledge. Prior to the invention of paper, palm leaves were most commonly utilized resources for encrypting messages and literature. These books have survived the centuries and are still highly valuable today. The elements that deteriorate palm leaf documents have been investigated, with their conservation strategy, using both ancient and modern approaches. Because palm leaf works are important for knowledge conservation, the research suggested that they be conserved as a first step. The research also suggested that the most essential task of today's archivists and libraries is to find efficient methods for the conservation of palm leaf works.

Rendering to Challa and Mehta [18], there are numerous businesses in India dedicated to protecting the earliest palm leaf scripts, owing to the importance of preserving the valuable texts of knowledge. Both natural and artificial processes influence palm leaves throughout time. With the advancement of technology worldwide, this research attempted to digitize palm leaf scripts required in a university library. One specific goal was to create an efficient method of palm leaf texts for efficient information retrieval. Segmentation, picture augmentation, processing, acquisition, and compression are only a few of the techniques available. All of these technologies use distinct algorithms that are effectively applied and produce the intended results. Given that ideal identification rates are not feasible with warped media and noise, selecting a proper image processing approach is important. This research focuses on image processing systems and algorithms utilized on palm leaf texts projected by many scholars for effective data recovery.

Vinoth et al. [19] investigated a method that aids in the conservation of palm leaves. The Tamil language has been identified as one of the world's classical languages. Tamil Nadu was discovered to be a location where palm leaf writings have been preserved. However, there are difficulties encountered with the protection of palm leaf writings. As a result, this research absorbed on the significance of conserving palm leaf work by converting it to digital text format. Digital gadgets are currently used for this resolution of conservation. This digital technology aims to accurately transform the characters and preserve the documents. Overall, the first step is to scan the palm leaf text and convert it to an image layout before saving it in a record. Following that, the pictures should be converted into a digital text format.

The major goal of Sonam and Poornima's [20] study was to create a system that allowed Tamil character identification from palm leaves, as well as caption through the captured pictures and preserving them for future use. Confident training devices have been carried out using a variety of approaches; however, the procedure of distinguishing the postures of Tamil characters is difficult. It is also worth noting that the Tamil language is considered complex compared to other languages due to the existence of curves, slopes, pits, and twists, resulting in variations in different writing styles. Many researches necessitate the adaptation of ancient Tamil characters to current characters to certify that the goal of developing computerized schemes for improving human knowing comprehension is increased. This suggested research is thought to be useful for segmenting Tamil characters and keeping them in an orderly folder, as well as for subsequent image processing. To enumerate the statistical characteristics of the segmented characters, GLCM matrix feature extraction is used. At this phase, utilizing GLCM characteristics, the segmented Tamil characters are distinguished from those in palm leaf manuscripts.

Convolutional neural networks can be used to recognize Tamil palm-leaf characters, as demonstrated by Sabeenian et al. [21]. Five layers of CNN were used in this study: convolution, pooling, activation, fully connected, and softmax classifiers. Scannable photographs of palm-leaf manuscripts were used to compile the database of character sets. There are 15 separate classes in the database, and each class has roughly 1000 samples. Generally speaking, CNN Classifier's recognition is determined to be between 96.1 and 100 percent. For each CNN layer, we extract a big quantum, resulting in an improved prediction rate.

## 3. Proposed Methodology

This section explains the workflow of the projected scheme, where the four major steps are included. The first step is the collection of cursive Tamil palm leaves scripts, followed by background removal, feature extraction, and classification as the further steps.  Figure 1 shows the workflow of the proposed methodology. The following section describes the significant things that are applied in the proposed model.

### 3.1. Dataset

The cursive Tamil palm leaf manuscripts are collected from the online images and stored in the database to document the target characters. In total, 100 images of cursive palm leaf texts are collected.  Figure 2 displays the sample collected cursive palm leaf texts. This data set is enhanced and experimented by different methods, which are represented in the following section.

### 3.2. Preprocessing

Digitized palm leaf manuscripts image has dark leaf color as background and text in the foreground. The presence of pickup noise in palm leaf manuscript images that happens while scanning or taking photo using the digital camera can either be reduced by sharpening or using any morphological methods. The sample image of the digital noise occurred image is shown in Figure 3. The noise removal is a necessary step to obtain useful information from digital text images. In preprocessing, the background has converted as black and foreground text as white in colors from the range of 0 to 255 into 0 and 1 only so that the characters are very clear and easy for processing. The background removal and morphological operations are the methods to promote the images to be suitable for text line segmentation. According to the shapes of the leaf, the images are processed by the morphological operations, where structuring element is applied to an input image and obtained the output image with same sizes. In MATLAB, a structuring element called strel is included for this operation, and finally, the output is obtained. By using this operation, noise and texture that are caused by simple thresholding are removed efficiently.

#### 3.2.1. Background Removal

In most of these systems, binarization is the scanned gray level image (labeling each pixel) print or background in document image analysis. Binarization is a process of assigning 0 s and 1 s using fixed threshold value. The fundamental idea of the fixed binarization method [21] is expressed in terms of relation. The background of palm leaf manuscripts can be taken as black by 0 and the foreground text as white by 1. Here, T shows global threshold value 50. After background removal, the preprocessed sample output image is shown in Figure 4(b) for the considered input image in Figure 4(a).

(1) $$\begin{array}{c} g\left(x,y\right)=\left\{\begin{array}{cc} 1, & \mathrm{if}\;f\left(x,y\right)\geq T,\\ 0, & \text{otherwise}, \end{array}\right. \end{array}$$

where “*x* and *y*” is an input image sampled from the input data distribution, and “*g*” is the ground truth image corresponding to the input image.

#### 3.2.2. Morphological Operations

In this operations, dilation and erosion are the fundamental operations. Addition of pixels with the boundaries of text objects in an image is known as dilation. Dilation is used to add pixels to the edges of regions or to fill in gaps in the image [22]. Erosion is the inverse of dilation. While dilatation raises the size of borders and fills holes, erosion diminishes the size of boundaries and enlarges holes. The reversal of this operation, i.e., extricating the pixels from the text object boundaries, is termed erosion [20]. In order to process the text-image in palm leaf manuscripts, the pixels may be added or removed depending on the size and shape of the text. In grayscale morphology, the images are mapped into the Euclidean space or grid ES ∪ {*r*, −*r*}, where the grayscale erosion of the palm leaf image *i* by text boundaries *b* is given as in the following relation:

(2) $$\begin{array}{c} \left(i\Theta b\right)=\int_{y\varepsilon B}^{\propto }\left[i\left(x+y\right)-b\left(y\right)\right]. \end{array}$$

### 3.3. Feature Processing

The text line segmentation in cursive Tamil palm leaf scripts is a Herculean task, and it influences till the end of the character recognition process. An absence of text line segmentation process is not possible for the successful character segmentation and character recognition in Tamil palm leaves. The TLS is applied on the preprocessed binary palm leaf text images to segment the text lines. The new way of approach in-text line segmentation of Tamil palm leaf images is to determine whether the obstacle is present between the text lines. Whenever the strokes of the character exceed from the text zone and extend in the space between the lines, then it is considered to be an obstacle in this case. The same is depicted in Figure 5.

#### 3.3.1. Space without Obstacle

The TLS, the text lines of Tamil palm leaf texts where the text line has enough space to the subsequent text lines or an elongation of character does not reach the below text line as in (Figure 6, are considered as space without obstacle or standard category. TLS can segment these text lines without any complication.

#### 3.3.2. Space with Obstacle

The presence of an obstacle in the space between the text lines can be categorized into two by the length of an obstacle that helps decide whether it is touching or overlapping text line. In Tamil character, an obstacle is an important part of deciding the character. The length of an obstacle that extends and reaches the subsequent text line is known as touching text lines (Figure 7). The first line character “யு/you/” is touching with the next line character “த/tha/”. In Tamil, the text line segmentation is complicated because if we ignore an obstacle of the character “யு”, it becomes “ய”, and if we cut an obstacle in a fixed length, the second line character “த/tha/” becomes “தி/thi/”. The overlapping text lines also have the same wrong prediction problem as touching text lines when we precede by existing text line segmentation algorithms. The proposed TLS solves the problem of touching and overlapping text lines by fixing the cutting edge at the end of an obstacle and also prevents wrong predictions of the character.

The purpose of text line segmentation is to precede the character segmentation. The touching and overlapping text lines complicate the text line segmentation and make the further process unproductive. An overlapping text line builds complication in-text line segmentation. An obstacle pervades the text zone of subsequent lines and mixed up with the character strokes that may precede wrong character prediction or different from expected character.

#### 3.3.3. Text Line Slicing (TLS)

The proposed TLS line segmentation algorithm identifies an extension of character strokes using four variables such as Vertical space (Vs), Horizontal space (Hs), Vertical Track (VT), and Horizontal Track (HT). The variable Vs used to count zeros vertically to know the stroke of a character exists in text line of binarized Tamil palm-leaf manuscript image. The total columns count of zeros is assigned to the variable VT and compared with the threshold. The value 1 denotes that the space has no obstacle, and 0 represents an obstacle. The variable Hs is used to count the zeros horizontally and the total value assigned to HT, and then, it is compared with a threshold value. Three values are used to decide whether an obstacle is present or not; zero (0) defines the space between the character in text line; one (1) defines that the character has an obstacle; and two (2) defines that the space is not found, which means that the character exists concurrently.

The obstacle creates touching text lines that can be defined by Connected Component (CC). The connectivity of the character is calculated by the weight of the character using CC. The touching and overlapping text line characters are considered single characters when they are connected to each other (Figure 8). An algorithm implementation (Figure 8(a)) proves obstacle identification in the space between the text lines, defines the category of connected characters by connected component, and calculates the weight for the character. When the minimum weight of the character identifies the TLS, the algorithm implements cutting edge (Figure 8(b)) to segment the connected text lines. Cutting edge is a breaking point of touching characters in text lines. The CC provides continuation of the character strokes and also vertical stroke values. The minimum value of the character stroke is known as the end of an obstacle that must be fixed as a cutting edge for the text lines. The sample images are shown in Figure 9.

### 3.4. Convolutional Neural Networks

Segmented and feature scaled images are given to the classifier model, which is CNN. Despite their popularity, ANNs were incapable of handling big datasets in recognition/classification responsibilities. To overwhelm these problems, profound learning is a new learning machine paradigm. It is a stacked, multilayered neural network. Earlier versions of the neural network, including the earliest perceptron, were superficial with one input and one output layer and a hidden layer between them. Each node layer in a deep-learning network trains on a range of features depending on the earlier layer output. An ideal will be well-organized if hidden layers can learn complex characteristics from seen data. Deep neural networks outperform previously unknown data. CNNs utilize a variant of the multilayer perceptron to meet the criterion of minimum preprocessing. CNNs are made up of an automated feature extractor and a trainable classifier with several layers, such as

- Convolutional Layer (CL),
- Pooling Layer (PL),
- Fully Connected Layer (FCL).

#### 3.4.1. CNN Architecture

CLs and PLs are used in basic CNN models, which offer a common architecture. CNNs apply a sequence of convolution operations on the input, with or without pooling and a nonlinearity activation function, and then send the output to the next layer. The CL employs filters (F) to extract important characteristics from the input picture for further processing. Each filter provides a unique property for accurate prediction. To maintain the image's size, the (zero padding) same padding is utilized; otherwise, its assistances decrease the sum of features. Each CL's convolutional output may be represented as

(3) $$\begin{array}{c} \text{Out}=\frac{\left(L_{\text{in}}+2\times \text{Pad}-F\right)}{S}+1, \end{array}$$

where *L*_*in*_ is identified as an input length, Out is identified as a length of the output, *S* is identified as a stride to filter slide, and Pad is identified as a padding.

A CL comprises generally 3-dimensional input (*H*_in_ × *W*_in_ × *C*_in_), where the height and width of the input are H_in_ and W_in_ and the channels of the input are C_in_. The calculation of the output function for each layer is exactly the same. The CLs produce parameters, neurons, and various connections, as mentioned earlier.

(4) $$\begin{array}{c} P=W_{t}+B, \end{array}$$

where *B* is a Bias, *W*_*t*_ is a weight of the CLs, and *P* is a parameter. A CL weight can be calculated as

(5) $$\begin{array}{c} W_{t}=C_{\text{out}}\times \left(H_{\text{in}}\times W_{\text{in}}\right)\times C_{\text{in}}, \end{array}$$

where *C*_out_ is output channels of the previous layer.

CLs and PLs are used in basic CNN models to offer a common architecture. CNNs use a succession of convolution operations to the input, coupled with/without pooling and a nonlinearity activation function, before sending the output to the subsequent layer. The filters (F) are used in the CL to extract important characteristics from the input picture for further processing. Each filter provides a unique property for precise estimate. To keep the picture size the same, identical padding (zero padding) is used; then, valid padding is used since its assistance decreases the sum of features. Each CL's convolutional output may be written as

(6) $$\begin{array}{c} W_{\text{out}}=\frac{\left(W_{\text{in}}-F\right)}{S}+1,\\ H_{\text{out}}=\frac{\left(H_{\text{in}}-F\right)}{S}+1, \end{array}$$

where *W*_out_ and *H*_out_ are height and width of the output, and *W*_in_ and *H*_in_ are height and weight of the input.

The weights and parameters change their values when data flows over a deep network, occasionally making the data too huge or too small. This is called the problem of the “interior covariate shift.” A modification in the distribution of the domain of a function is called a covariate shift. Each layer entry is affected in deep networks by its parameters, which means that a slight network change can affect the whole network. Such internal layer modifications may cause the deep network to experience an internal covariate shift issue. This problem is generally overcome by normalizing the data in each mini-batch. The general formulae of Batch normalization (BN) are presented in the next section. It is used to allow every network layer to do learning more independently and used to normalize the output of the previous layer. In addition, overfitting is minimized, because it has a slight regularization effect. BN operates on 4D inputs, which may be represented as a small batch of 3D inputs. During training, this layer retained a running evaluation of its calculated mean and variance with a momentum of 0.1.

(7) $$\begin{array}{c} \mu \left[x_{i}\right]=\frac{1}{n}\sum_{i=1}^{n}x_{i}, \end{array}$$

where *μ*[*x*_*i*_] is the mini-batch mean value, *x*_*i*_ is represented as the value of the mini-batch elements, and

(8) $$\begin{array}{c} \sigma^{2}\left[x_{i}\right]=\frac{1}{n}\sum_{i=1}^{n}{\left(x_{i}-\left[x_{i}\right]\right)}^{2}, \end{array}$$

where *σ*[*x*_*i*_] is the mini-batch variance values:

(9) $$\begin{array}{c} {\hat{x}}_{i}=\frac{x_{i}-\mu \left[x_{i}\right]}{\sqrt{\sigma^{2}\left[x_{i}\right]}}+\epsilon , \end{array}$$

where ${\hat{x}}_{i}$ is the mini-batch normalization:

(10) $$\begin{array}{c} Y_{\text{out}}=\gamma {\hat{x}}_{i}+\beta , \end{array}$$

where *Y*_out_ is the mini-batch normalized value, and *γ* and *β* are the learnable parameters:

(11) $$\begin{array}{c} f\left(x\right)=\max\left(x,0\right), \end{array}$$

where *f*(*x*)  denotes the nonlinear activation function. The goal of FCL is to use the characteristics of the CLs and PLs to classify pictures into distinct classes based on the training dataset.

As previously mentioned, a computationally simple and efficient cursive character specific neural network system is the aim. To accomplish this, a six-layer architecture is proposed, with each layer essentially including CL > Batch Normalization (BN) > ReLU > Max Pooling Layer (Max-PL) (see Figure 10). PLs are employed in the projected model to lower the spatial dimensions, which implies that they will lessen the number of parameters inside the model, with a process known as downsampling or subsampling. Following each PL layer, BN is employed to deal with the interior covariate shift difficult. As the network becomes deeper, it may become trapped in the saturation area, resulting in a vanishing gradient issue/problem. To address this, the planned network employs Rectified Linear Unit (ReLU). The complex patterns in the input data are learned by the network using activation function, and ReLU is considered as an activation function in this model, where it does not activate all the neurons at the same time. The goal of FCL is to use the convolutional and PL features to categorize the input picture into multiple classes depending on the training dataset.

The subsections that follow provide a brief explanation of the suggested CNN model construction.

*(1) ThimuNet Architecture*. In the preceding sections, a fundamental introduction of CNN architecture was presented. This section discusses the proposed CNN architecture “ThimuNet,” which is meant to identify handwritten cursive characters. The goal is to create a CNN model that can learn differentiating features for handwritten character identification in a fraction of the time and space required by present models. Figure 10 depicts ThimuNet's architecture, which consists of six levels. The input image has a resolution of 64*∗*64 pixels. First, the supplied image is scaled to (64*∗*64) pixels in size. The first layer then receives picture pixels as input. Each CL alternates with a subsampling or pooling layer, which takes the pooled maps as input.

CL, Max-PL, and FCL are denoted as *C*_*x*_, *M*_*x*_, and *FC*_*x*_ correspondingly, in the following discussion, where *x* is the layer index. The input for the first CL, C1, will be  64 × 64 × 1. The output of C1*∗*(“C” after numerals represents layer number), ReLU, and batch normalization is applied. As a consequence, 22 subsampling processes were performed. *M*_2_ is a max-PL with 32 feature maps of 32 × 32 dimensions.  Table 1 shows the calculation of trainable characteristics and trainable links. The C3 layer has 64 feature maps. C3's output feature maps are linked to M4. ReLU and BN are implemented after each CL layer. C5, C7, and C9, like the previous convolutional layers, convolute the prior feature maps. Max-PLs are linked to each subsequent CL.

The output volume will be 512 (2 × 2 × 512) after the final layer. As a result, they can extract characteristics that are more resistant to local changes of the input pictures. This FC layer has been flattened to 1 × 1 × 2048, used to compute the class scores. This entire layer scheme is similar to a conventional feedforward network by overlapping the map element and kernel element input on each specific layer and adding results together for the output to that particular layer after calculation. Gradients of error have been calculated via backpropagation. Gradient descent was employed to update all network weights (equation (5)) and parameter values (equation (4)) to reduce output errors. A concise architectural indication is as follows: 32*C*1 − BN − RELU − 2*P*2 − 64*C*1 − BN − RELU − 2*P*2 − 128*C*1 − BN − RELU − 2*P*2 − 256*C*1 − BN − RELU − 2*P*2 − 512*C*1 − BN − RELU − 2*P*2 − 2048FC OUTPUT.where XC*y* denotes a *CL* with a total of *X* kernels and a stride of *y* pixels in this representation, *MP n* signifies a Max-PL 8 with a *M*  ×  *M* pooling window and a stride of *n* pixels, BN signifies a Batch normalization 18, and *NFC* signifies a *FC* layer with *n* neurons.

## 4. Results and Discussion

As previously stated, the objective of this study is to provide a superior CNN model than the current models for the gathered cursive dataset. To build the suggested neural network design, PyTorch7 was used as the Python-based framework. On these gathered datasets, evaluation of many modern models such as LeNet5, ResNet (18/34/50), AlexNet, DenseNet121, InceptionNet v3, and others was also conducted to have a comparative analysis. All of these trials are carried out on a system equipped with Intel Core i3 CPUs, 16 GB of RAM, and an NVIDIA graphics card with 4 GB of internal memory and 768 CUDA cores.

### 4.1. Result Evaluation of Proposed ThimuNet

This section validates the proposed CNN performance with other techniques in terms of various parameter metrics. The major parameters such as Precision, Balanced Classification Rate (BCR), Recall, Sensitivity, Misclassification Penalty Metric (MPM), Specificity, Balanced Error Rate (BER), F-measure based on sensitivity and specificity, Peak Signal to Noise ratio (PSNR), and Distance Reciprocal Distortion (DRD) can be computed for the Tamil Palm leaf manuscripts. However, in this work, only a few parameters are considered for the validation process; the reason is that it is a collected cursive Tamil Palm Leaf manuscript and cannot apply all major parameters.

(12) $$\begin{array}{c} \text{Accuracy }=\frac{\left(xp+xn\right)}{\left(xp+yp+xn+yn\right)},\\ \frac{\text{Recall}}{\text{Sensitivity}}=\frac{xp}{\left(xp+yn\right)},\\ \text{Precision }=\frac{xp}{\left(xp+yp\right)},\\ F1-\text{Measure }=2\frac{\text{Precision }\times \text{Recall}}{\text{Precision}+\text{Recall}}, \end{array}$$

where *xp* is denoted as True positive, *xn* is denoted as true negative, *yp* is described as false positive, and *yn* is represented as false negative.

The reason for comparing various pretrained models on CNN is that they are significantly more accurate than the custom-built model of CNN. In addition, the pretrained models can effectively train on large datasets and directly use the weights and architecture obtained to detect the cursive characters of Tamil on palm leaves. LeNet is the base for all ConvNets, which is mainly used for detecting the handwritten characters. ResNet is used to solve the vanishing gradient problem by making the CNN to construct with more than thousands of convolution layer without the increase of training error percentage and outperform the shallower networks. AlexNet is developed by using eight layers with learnable parameters, which has the ability to leverage GPU for training and being able to train with vast numbers of parameters. In DenseNet, each layer is connected to every other layer, and it also alleviates the vanishing gradient problem. Moreover, the features are reused in this model, feature propagation is strengthened and minimized the number of parameters. Initially, the proposed CNN performance is validated with the existing technique in terms of PSNR and BER [23], tabulated in Table 2 and Figure 11.

The performance of the technique is improved when the PSNR level is high and BER is low. For instance, LeNet and AlexNet have low PSNR values (5.77 and 7.08), whereas ResNet and DenseNet achieved nearly 16 of PSNR. But the proposed ThimuNet achieved 17.74 of PSNR. The existing techniques such as LeNet and AlexNet achieved high BER (i.e., nearly 28.5), where ResNet and DenseNet achieved 11.9 and 7.52 of BER. The proposed ThimuNet achieved very low BER, i.e., 6.06, when compared with other existing techniques. The reason is that the proposed ThimuNet is well adapted with all input features.  Table 3 and Figure 12 show the experimental results of proposed ThimuNet on precision, recall, sensitivity, specificity, and F-measure.

In the precision experiments, the LeNet achieved 63%, AlexNet achieved 84%, ResNet achieved 91%, and DenseNet achieved 94%, but the proposed ThimuNet achieved only 92%. The reason is that some features are wrongly classified, and some collected cursive writings are not properly removed by using preprocessing techniques. After that, recall and sensitivity experiments are carried out to validate the performance of the proposed ThimuNet. The existing technique LeNet achieved 65%, ResNet achieved 79%, AlexNet achieved 47%, and DenseNet achieved 86%, whereas the proposed ThimuNet achieved 89% recall and sensitivity. This proves that the proposed net achieved better performance than existing techniques. Finally, specificity and F-measure experiments are performed. All the existing techniques achieved nearly 85% to 90% of F-measure and 93% to 99% of specificity, where the proposed ThimuNet achieved 90.51% of F-measure and 99% of specificity.  Table 4 and Figure 13 provide the comparative analysis of proposed ThimuNet with existing techniques in terms of accuracy.

The above table and Figure clearly prove that the proposed ThimuNet achieved higher performance than existing techniques in terms of accuracy. For example, the LeNet achieved 71% accuracy, ResNet achieved 88% accuracy, AlexNet achieved 66% accuracy, DenseNet achieved 92% accuracy, and the proposed ThimuNet achieved 94% accuracy. Finally, the prediction time of proposed ThimuNet for classifying the cursive Tamil Palm Leaves Manuscript is given in Table 5 and Figure 14.

The existing LeNet, AlexNet, and ResNet prediction time achieved nearly 1.08 seconds, while the DenseNet achieved 0.95 seconds for the classification. However, the proposed ThimuNet achieved less prediction time (0.80 seconds) than existing techniques. The proposed ThimuNet achieved better performance from all experimental analysis and classified wrong cursive letters due to irrelevant features. This problem can be solved by incorporating efficient feature selection techniques with proposed ThimuNet.

## 5. Conclusion

Tamil is the world's oldest languages and has attainment popularity among scholars throughout the world due to its historical relevance and capacity to persist for centuries. Individual interests and ideologies of academics have shaped study on palm leaves manuscripts in Tamil literature over the periods and in a variety of ways. The most prevalent topic of research in the actual world is cursive character recognition of ancient Tamil characteristics, and it focuses on the documentation of Tamil characters to guarantee that a large amount of data is gathered. However, due to improper care, palm leaf manuscripts have been destroyed, as numerous people held them by default. As a result, a rigorous examination of Tamil palm leaf texts, translation, and cataloguing of their publishing were necessary. Thousands of palm leaf manuscripts exist in the hands of institutes and separate healers, but they must be digitized, and proper catalogues are developed for the future. Similarly, numerous researches on the cursive handwriting recognition of the Tamil language are included in the survey. There is, however, no universal technique for identifying cursive Tamil letters (with sufficient accuracy) in their whole. As a result, various approaches have been used in each stage of the recognition process.

This work is one of the first attempts to build cursive training datasets by manual and automated segregation of Tamil palm leaf scripts. Future researchers could use the data set to develop expert systems that could then be used for a range of purposes, such as a character classification based on the century they have evolved and the identification of extinguished characters, and the identification of characters whose shape could have changed. The research attempted to segregate ancient Tamil palm leaf scripts to produce a massive amount of Tamil cursive character information. There have been no previous investigations on the identification of cursive characters in Tamil palm leaf scripts. The ThimuNet of CNN is used in this research project to classify cursive Tamil characters, and its performance is confirmed. In order to improve the performance of proposed model, the weight of the input parameters must be optimized, which is considered as future scope of this research model. In addition, preprocessing plays a major role in removing unwanted cursive writings; therefore, an effective preprocessing technique is implemented along with the developed model for better performance.

## Figures and Tables

**Figure 1:** Working procedure of proposed methodology.

**Figure 2:** Sample cursive Tamil palm-leaf manuscript.

**Figure 3:** Sample noise occurred image before preprocessing.

**Figure 4:** Preprocessed sample output image. (a) Input image. (b) Background removal. (c) Morphology.

**Figure 5:** Sample obstacle.

**Figure 6:** Some of the sample text lines. (a) No obstacle, (b) obstacle not reached to the below text line.

**Figure 7:** Sample obstacle defined in the text line.

**Figure 8:** Sample text line slicing. (a) Implementation on Tamil palm-leaf manuscript, (b) cutting edge.

**Figure 9:** Illustration of the unique palm-leaf manuscript representing characters attained as an output with the typescripts.

**Figure 10:** Proposed modified CNN architecture—ThimuNet.

**Figure 11:** Graphical representation of proposed ThimuNet in terms of PSNR and BER.

**Figure 12:** Performance analysis of proposed ThimuNet with existing techniques.

**Figure 13:** Graphical representation of proposed ThimuNet in terms of accuracy.

**Figure 14:** Comparative analysis of proposed ThimuNet in terms of prediction time.

**Table 1:** Summarization of different parameters of the proposed ThimuNet.

Convolutional layer	Parameters	Neurons	Connections	Activations
Layer 0- INPUT (64 × 64) 3 channels	0	0	0	64 × 64 × 3 *A* = 12,288
Layer 1- FILTER (5 × 5) 32 outputs	Wt = 32 × (5 × 5) × 3 *B* = 32 *P* = (2400 + 32) = 2,432	(64 × 64) × 32 *N* = 1,31,072	*C* = 32,76,800 (64 × 64) × 32 × (5 × 5)	Conv = 64 × 64 × 32 pool = 32 × 32 × 32 BN = 64 × 64 × 32 *A* = 294,912
Layer 2- FILTER (5 × 5) 64 outputs	Wt = 64 × (5 × 5) × 32 *B* = 64 *P* = (51200 + 64) = 51,264	(64 × 64) × 64 *N* = 2,62,144	(64 × 64) × 64 × (5 × 5) *C* = 65,53,600	Conv = 32 × 32 × 64 BN = 32 × 32 × 64 pool = 16 × 16 × 64 *A* = 147,456
Layer 3- FILTER (5 × 5) 128 outputs	Wt = 128 × (5 × 5) × 64 *B* = 128 *P* = (204800 + 128) = 2,04,928	(64 × 64) × 128 *N* = 5,24,288	(64 × 64) × 128 × (5 × 5) *C* = 1,31,07,200	Conv = 16 × 16 × 128 BN = 16 × 16 × 128 pool = 8 × 8 × 128 *A* = 73,728
Layer 4- FILTER (5 × 5) 256 outputs	Wt = 256 × (5 × 5) × 128 *B* = 256 *P* = (819200 + 256) = 8,19,456	(64 × 64) × 256 *N* = 10,48,576	(64 × 64) × 256 × (5 × 5) *C* = 2,62,14,400	Conv = 8 × 8 × 256 BN = 8 × 8 × 256 pool = 4 × 4 × 256 *A* = 36,864
Layer 5- FILTER (5 × 5) 512 outputs	Wt = 512 × (5 × 5) × 256 *B* = 512 *P* = (3276800 + 512) = 32,77,312	(64 × 64) × 512 *N* = 20,97,152	(64 × 64) × 512 × (5 × 5) *C* = 5,24,28,800	Conv = 4 × 4 × 512 BN = 4 × 4 × 512 pool = 2 × 2 × 512 *A* = 18,432
Fully connected layer (FC layer)—46 class outputs	Wt = 512 × (2 × 2) × 46 *B* = 46 *P* = 94,208	0	0	*A* = 46

**Table 2:** Validated results of proposed model with existing techniques.

Network type	PSNR	BER
LeNet	5.77	28.42
ResNet	15.69	11.9
AlexNet	7.08	29.74
DenseNet	16.08	7.52
ThimuNet	17.74	6.06

**Table 3:** Experimental results of proposed ThimuNet with existing techniques.

Network type	Precision (%)	Recall (%)	Sensitivity (%)	Specificity (%)	F-measure (%)
LeNet	63	65	65	79	63.87
ResNet	91	79	79	99	85.01
AlexNet	84	47	47	93	57.45
DenseNet	94	85	86	99	90.14
ThimuNet	**92**	**89**	**89**	**99**	**90.51**

**Table 4:** Comparative analysis of proposed ThimuNet on the basis of accuracy.

Network type	Accuracy (%)
LeNet	71
ResNet	88
AlexNet	66
DenseNet	92
ThimuNet	**94**

**Table 5:** Prediction time of proposed ThimuNet for classification of cursive Tamil palm leaves manuscript.

Network type	Prediction time (s)
LeNet	1.06
ResNet	1.09
AlexNet	1.04
DenseNet	0.95
ThimuNet	0.80

## Data Availability

The data used to support the findings of this study are available from the corresponding author upon request.
